The article "The Photocatalytic Effects of Modified Hydrothermal Nanotitania Extraction on the Skin and Behavior of Sprague-Dawley Rats" was published in 2021. Journal: Biomed Res Int.

# The Photocatalytic Effects of Modified Hydrothermal Nanotitania Extraction on the Skin and Behavior of Sprague-Dawley Rats

**DOI:** 10.1155/2021/6173143

**Published:** 2021-11-23

**Authors:** Ahmad Mukifza Harun, Huzaika Awang, Nor Farid Mohd Noor, Nur Mohamad Makhatar, Mohamad Ezany Yusoff, Nor Dalila Nor Affandi, Mohammad Khursheed Alam

**Affiliations:** ^1^Engineering Faculty, Universiti Malaysia Sabah, Jalan UMS, 88400 Kota Kinabalu, Sabah, Malaysia; ^2^Pusat Persediaan Sains dan Teknologi, Universiti Malaysia Sabah, Jalan UMS, 88400 Kota Kinabalu, Sabah, Malaysia; ^3^Faculty of Medicine, Universiti Sultan Zainal Abidin (UniSZA), Medical Campus, Jalan Sultan Mahmud, 20400 Kuala Terengganu, Terengganu, Malaysia; ^4^School of Dental Sciences, Universiti Sains Malaysia, Health Campus, 16150 Kubang Kerian, Kelantan, Malaysia; ^5^Textile Research Group, Faculty of Applied Sciences, Universiti Teknologi MARA, Shah Alam 40450, Malaysia; ^6^College of Dentistry, Jouf University, Sakaka 72721, Saudi Arabia; ^7^Department of Dental Research Cell, Saveetha Dental College and Hospitals, Saveetha Institute of Medical and Technical Sciences, Chennai, India

## Abstract

**Background:**

Potential antibacterial substances, such as titanium dioxide (TiO_2_), are being extensively studied throughout the research world. A modified hydrothermal nanotitania extraction was shown to inhibit *Staphylococcus aureus* growth in the laboratory. However, the toxicity effect of the extract on rats is unknown. In this study, we observed the effects of a modified hydrothermal nanotitania extraction on the skin and behavior of Sprague-Dawley rats.

**Methods:**

Sprague-Dawley (*Rattus norvegicus*) rats were used as the experimental animals. The skin around the dorsum of the tested animals was shaved and pasted with 0.1 mg and 0.5 mg of the nanotitania extraction. The color and condition of the pasted area and the behavior of the animals were observed.

**Results:**

0.1 mg nanotitania extraction application on the dorsum of the rat produced no skin color changes at day 1, day 3, day 5, or day 7 postapplication. There were no changes in their behavior up to day 7 with no skin rashes or skin scratches seen or fur changes. However, 0.5 mg of nanotitania extraction resulted in redness and less fur regrowth at day 7.

**Conclusions:**

A 0.1 mg modified nanotitania extraction was observed to have no effect on the skin of Sprague-Dawley rats.

## 1. Introduction

In the health and medical sector, the bacteria most widely recognized as a skin host and infector of soft tissue is *Staphylococcus aureus* (*S. aureus*) [1]. It is the principal organism associated with catheter-related infections, such as infective endocarditis—a devastating heart condition [2]. *Staphylococcus aureus is* the main reason for surgical operative infections and postoperative complications in the operating theatre (OT) and clinical settings [3]. Bacterial infection in the blood or septicemia is potentially fatal and related to *S. aureus*. In short, *S. aureus* is one of the most prevalent components in hospital-acquired bacteremia [4]. Long-term illnesses connected with the *S. aureus* infections are respiratory infections such as pneumonia, contagion in the bones, and joint infections. Besides the *S. aureus* associated with hospital infections, a strain of methicillin-resistant *Staphylococcus aureus* (MRSA) requires intensive treatment [5]. The main sources of *S. aureus* bacteria are the nasal cavity and throat [6]. In certain medical fields like pediatrics [7], *S. aureus* is one reason why children end up in wards with respiratory symptoms, typically associated with cystic fibrosis [8].

The article "The Photocatalytic Effects of Modified Hydrothermal Nanotitania Extraction on the Skin and Behavior of Sprague-Dawley Rats" was published in 2021. Journal: Biomed Res Int.

Titanium dioxide (TiO_2_) has been extensively researched due to its potential as an antibacterial substance. One study has shown that increasing the density of TiO_2_ nanoparticles has been known to bring down the replication t rate of bacteria such as *Escherichia coli* [9]. Furthermore, Martinez-Gutierrez et al. have found that the accumulation of TiO_2_ with other potential substances such as silver can lead to antimicrobial action [10]. In addition, synthesized TiO_2_ nanoparticles from an extraction of the *Psidium guajava* aqueous leaf displayed an antibacterial event on *S. aureus*, *Pseudomonas aeruginosa*, *E. coli*, and *Proteus mirabilis* [11]. In previous research, the authors determined that modified hydrothermal nanotitania has the potential to control the growth of *S. aureus* in the microbiology lab [12]. This paper investigates the toxicity effects related to the photocatalytic properties of TiO_2_. According to Miao et al., titanium dioxide (TiO_2_), iron oxide, copper oxide, and zinc oxide are semiconductors that have been extensively studied as photocatalysts due to their wide absorbance range [13]. Because of its long durability, chemical and optical stability, strong oxidizing properties, nontoxicity, low cost, and transparency to visible light [14], TiO_2_ has been used in many photocatalytic applications and is considered the most effective photocatalyst.

The photoactivity of a photocatalyst depends on the rate of photogenerated electrons in the conduction band (CB) by light absorbance and the formation of holes in the valence band (VB) [15].  Figure 1 shows the overall of the general photocatalysis process. The wavelength response in TiO_2_ needed to generate electrons in CB is limited to the light in the UV region (10–400 nm) due to its relatively large bandgap (3.0–3.2 eV) [16]. In addition, the lifetime of the electron hole pair required to perform the oxidation and reduction reactions is very short and the electron hole can be recombined within a few nanoseconds [17]. As a result, several studies have been conducted to determine a way to extend the wavelength responses and overcome recombination rate issues. According to Mohammad et al., modifying the TiO_2_ structure in the form of nanotitania, nanotubes, nanomembranes, nanofilms, and other structures will increase surface area and electron hole pair active sites and be a tunable structural property that can act as an excellent catalyst in various applications [13, 18]. Numerous modifications to the TiO_2_ structure have been implemented, including doping with metal and nonmetal ions, dye sensitization, and semiconductor coupling [17]. Due to the antibacterial properties of TiO_2_ and the significance of silver in medical applications, silver-doped titania has been regarded as a potential photocatalyst in various applications. It is mainly used in the manufacture of coated sanitaryware, medical instruments, food preparation surfaces, and air conditioning filters among others [13]. According to Choi et al., silver can trap electrons from TiO_2_ and leave holes for organic species degradation reactions [19]. In addition, the ability of silver to extend the wavelength response in nanotitania towards ultraviolet has been successfully shown [19]. The silver in nanotitania promotes the phase transformation from anatase to rutile, which enhances its surface area and electron hole pairing and improves its photoactivity performance [17].

The article "The Photocatalytic Effects of Modified Hydrothermal Nanotitania Extraction on the Skin and Behavior of Sprague-Dawley Rats" was published in 2021. Journal: Biomed Res Int.

Previous studies by the authors have shown some promising results with modified hydrothermal TiO_2_ extraction [7, 20, 21], including demonstrating its ability to eradicate respiratory bacteria and fungus through self-disinfection [12, 22, 23]. Previous experiments with nanotitanium dioxide have also resulted in the suppression of its mutagenic capability [23] and its toxicological properties [24, 25]. Other results of manipulating the photocatalytic properties have been the development of dye-sensitized solar cells [26, 27]. The photocatalytic effect has been reported in the nanotitania ability to eradicate the growth of *Klebsiella pneumoniae* and *Haemophilus influenzae* [28].

From previous results, the authors concluded that this substance has the potential to inhibit the growth of bacteria in the real world. It was decided to first test the extraction on an animal skin. In this study, the effects of modified hydrothermal nanotitania extraction (attributed to the photocatalytic properties of TiO_2_) on the skin and behavior of Sprague-Dawley rats were observed.

The article "The Photocatalytic Effects of Modified Hydrothermal Nanotitania Extraction on the Skin and Behavior of Sprague-Dawley Rats" was published in 2021. Journal: Biomed Res Int.

## 2. Materials and Methods

This test is aimed at documenting the effect of modified hydrothermal nanotitania on rat skin and physical and behavioral changes of the rats after having the substance pasted on their bodies. Male and female Sprague-Dawley (*Rattus norvegicus*) rats (20 rats) aged between 10 and 12 weeks and weighing 250 g–400 g were chosen. Sprague-Dawley rats were chosen because of their availability in the lab. The animals were maintained with a twelve-hour light/dark cycle at room temperature and kept in polypropylene cages with access to a standard pellet diet and water *ad libitum.* The rats were maintained with a twelve-hour light/dark cycle at room temperature and were kept in polypropylene cages consisting of 3 rats per cage. In this experiment, 20 rats were used, which was divided into three groups: 10 rats for the control and another 10 rats for the skin test (5 rats for 0.1 mg and 5 rats for 0.5 mg nanotitania extraction).

The rats had been acclimatized by daily body weight measuring for 5 days. Their skin was shaved at the dorsum using a hair shaver. The shaved area was pasted with a modified nanotitania extraction of 0.1 mg in a dilution with saline water, while a control substance was pasted on the control rat's skin. The extract was pasted at the right side of the shaved area to compare the reactions at both the applied and nonapplied sites of the same animal. The paste was applied directly to the skin without mixing to make sure that the maximum effect could be observed and to avoid bias caused by contact with other substances. Changes to the skin were observed on day 1, day 3, day 5, and day 7. The researchers looked out for any color changes in the shaved skin area, behavioral changes, such as being restlessness in the cage, or changes in eating behavior. Any skin reactions (e.g., rashes) or scratch marks were noted, and photos were taken on alternate days in accordance with the observation schedule. The same test was repeated with another group of rats using 0.5 mg of modified nanotitania extraction. The control rat group is the shaved dorsum of the rat without any substance pasted on it.

This experiment was reviewed and approved by Universiti Sains Malaysia (USM) Institutional Animal Care and Use Committee (USM IACUC) USM/IACUC/2019/(121)(1041). This test was conducted in Universiti Sains Malaysia.

## 3. Results

The condition of the rats and their skin of the shaved site was observed on alternate days in accordance with the test schedule. The results are presented in a table for easy evaluation. Our application of 0.1 mg nanotitania extraction on the dorsum of the rats produced no skin color changes such as reddening or darkening at day 1, day 3, day 5, or day 7 postapplication (Table 1). No skin rashes were noted throughout the observation period. The rats displayed no changes in their behavior (daily food consumption/eating and movement routine in the cage) up to day 7. Furthermore, no skin rashes or scratches or changes to the condition of the fur were noted (Table 1). Similar regrowth of fur at the shaved site was evident at days 2 and 3 postapplication. A photo of the shaved area after the application of the substance at the rat dorsum is shown in Figure 2.

The article "The Photocatalytic Effects of Modified Hydrothermal Nanotitania Extraction on the Skin and Behavior of Sprague-Dawley Rats" was published in 2021. Journal: Biomed Res Int.

In contrast, the application of 0.5 mg nanotitania extraction on the dorsum of rats resulted in skin color changes observed at day 1, day 3, day 5, and day 7 postapplication (Table 2). Redness of the skin was noted, especially at the site of the application. The fur at the shaved site (application site) also showed reduced growth compared to that at the nonapplied site. However, the rats displayed no changes in their behavior (eating and movement) and no skin rashes or skin scratches were evident throughout the observation window. The photo of the shaved area or dorsum of the rat is shown in Figure 2 comparing with the control rat group. Noted that histopathological evaluation was not done in this study as the aim is at detecting any gross changes over rat the skin.

## 4. Discussions

The aim of this test was at checking the reaction of the modified nanotitania extraction with the skin of the rats. The fur at the dorsum of the animal was shaved, and the substance was directly applied on to it at the right side of the shaved area, while the left side of the shaved area was left undisturbed to make sure that direct comparison could be made. The behavior of the animals was also observed, specifically their eating and movement patterns inside the cage. The growth and condition of the fur throughout the observation were also noted. The nanotitania extraction produced no skin changes after application of 0.1 mg of the substance on the dorsum of the skin. No skin color changes were seen. The fur regrew normally at the shaved area. The rats' behavior did not change in terms of movement and eating habits up to day 7. The animals' skin displayed no reactions to the applied substance, such as scratch marks or rashes. It appears that 0.1 mg substance has no effect on the skin and produces no animal reaction. The animal may not realize that the substance has been applied as no behavioral changes were seen. It is therefore suggested that 0.1 mg is safe for application to the mammalian skin, specifically that of rats.

The article "The Photocatalytic Effects of Modified Hydrothermal Nanotitania Extraction on the Skin and Behavior of Sprague-Dawley Rats" was published in 2021. Journal: Biomed Res Int.

In contrast, 0.5 mg of the substance resulted in skin color changes, i.e., redness at the applied site. No scratch marks or rashes were seen and no reaction was observed from the rats in terms of daily behavior. Although the rats may not have noticed the application of the substance, skin change was observed at the shaved site.

Consequently, it is not recommended that the substance be applied beyond 0.1 mg as it may affect the skin color, although it is unlikely to cause rashes or reactions such as scratching.

This experiment was scheduled after our modified nanotitania extraction was found to inhibit the growth of *Staphylococcus aureus* in our microbiology lab [14]. The ability of this substance to prevent the growth of *S. aureus* shown its potential to be used as an antibacterial substance. *S. aureus* is one of the main bacteria causing many health problems in human specifically skin-related problem. This experiment shows the probable function of this substance as a physical barrier for bacterial growth in the next step of the study. The histopathological test was not done in this test as the initial aim is to see the gross changes over the rat skin as other experiments which histopathological test is essential [15]. In addition, we found that this substance was not nontoxic to the cells [16] and noncarcinogenic [17].

## 5. Conclusions

No skin or behavioral changes were evident in the laboratory specimens after applying the 0.1 mg modified nanotitania extraction. It is noted that our extraction of nano-TiO2 by the hydrothermal process caused a photocatalytic reaction to occur that does not harm the skin of rats or alter their behavior.

## Figures and Tables

**Figure 1:** General photocatalysis process.

**Figure 2:** The reaction to the substance on the skin as observed on day 7. (a) Normal skin appearance of the control rat group. (b) Skin color changes (redness) were observed after 0.5 mg was pasted on the dorsum of the rat. The dorsum appeared to have less fur growth on the side of the applied substance.

**Table 1:** Testing the rat skin with 0.1 mg modified nanotitania extraction.

Skin observation/days	Day 1	Day 3	Day 5	Day 7
Color changes	No	No	No	No
Animal behavior	Normal	Normal	Normal	Normal
Skin rashes	No	No	No	No
Skin scratches	No	No	No	No
Fur changes	No	No	No	No

**Table 2:** Testing the rat skin with 0.5 mg modified nanotitania extraction.

Skin observation/days	Day 1	Day 3	Day 5	Day 7
Color changes	Yes	Yes	Yes	Yes
Animal behavior	Normal	Normal	Normal	Normal
Skin rashes	No	No	No	No
Skin scratches	No	No	No	No
Fur changes	Yes	Yes	Yes	Yes

## Data Availability

All data are available within the manuscript.
